# Digital Twins Model of Industrial Product Management and Control Based on Lightweight Deep Learning

**DOI:** 10.1155/2022/4452128

**Published:** 2022-03-24

**Authors:** Zuoyue Huang, Zhitao Yan

**Affiliations:** School of Engineering and Architecture, Chongqing University of Science and Technology, Chongqing 401331, China

## Abstract

Digital twins (DTs) can realize the integration of information and entities. It is widely used because of its simulation characteristics and virtual reality (VR) mapping. Its application to industrial product management and control is explored. First, the concept and the functions in different stages of DTs are expounded. Second, the Workench simulation platform and SolidWorks software are applied in the design of the aluminum alloy flange according to DTs in the design stage of industrial product management and control. Third, the role of DTs in industrial product management and control is confirmed through a comparative experiment. Finally, an intelligent algorithm for the automatic identification of internal defects is designed based on lightweight deep learning to improve the efficiency of ultrasonic detection. The results show that the accuracy of the lightweight convolution neural network (CNN) is 94.1%; the model size is 2.9 MB; the network is more lightweight and has an excellent performance in ultrasonic defect detection; the nonlinear finite element analysis results and the test results are consistent. Therefore, it is proved that the finite element analysis method is reliable and helps to improve the efficiency and shorten the design cycle. The emergence of DTs provides a technical scheme for product management and control under the three-dimensional model.

## 1. Introduction

In recent years, with the continuous development of new technologies such as artificial intelligence (AI) and the Internet of things (IoT), which have been applied to the manufacturing industry one after another, a large number of industrial applications under the condition of new technologies have also emerged one after another and have attracted the attention of all countries. In the *Made in China 2025* plan, China government proposes that intelligent manufacturing will become an important direction and core content of China's industrial development in the future [1]. Intelligent manufacturing is a system integrating intelligence and man-machine integration. Concurrently, it can also carry out a series of intelligent activities in the process of manufacturing [2].

The key problem of intelligent manufacturing is how to integrate the physical world and the information world, and the DTs just solve this problem [3]. So far, DTs have been successfully applied to different industries, including product design, production, prediction, health management, and some other fields [4, 5]. DTs make full use of the physical model, sensor update, and operation history, and other data integrate multidisciplinary, multiphysical quantity, multiscale, and multiprobability and complete the mapping in the virtual space, to reflect the simulation process of the whole life cycle process of corresponding physical equipment. Furthermore, it can also realize some scenarios such as real-time monitoring, data collection, simulation, analysis, and reasoning of physical objects [6–11]. In the process of continuous improvement and development of the concept of DTs, academia has mainly carried out relevant research on the modeling, the integration of information physics, interaction and collaboration, and service applications of DTs. At present, some research has been carried out on the framework and modeling process of DTs modeling, but there is no consistent conclusion. Some progress has been made in modeling theory, including physical behavior research, nondestructive material measurement technology, quantitative error, and confidence evaluation. These auxiliary technologies will help to determine the model parameters, construct the behavior constraints, and verify the model accuracy. Using the DTs model for personalized production of products and integrating the DTs model into the product design and production process can achieve rapid product design and improve production efficiency and realize personalized product customization, modular design, and highly scalable production. In ultrasonic testing technology, identifying and classifying the defects of the detected object is exactly the application category of pattern recognition. At present, the most commonly used method in ultrasonic testing is neural networks. The neural network has good adaptability and can learn and form many complex judgment models in mode space. However, its application in practical engineering is limited due to its poor stability. With the progress of computer vision, it also further promotes the development of ultrasonic detection technology. The convolutional neural network (CNN) shows great advantages in image recognition and classification. With the help of computer vision, the detection efficiency and the quality of detection results will be greatly improved. In the existing CNN, the deeper the network is and the more the number of feature planes is, the larger the feature space the network can represent and the more the network can learn. However, the CNN model will become more and more complex if its performance is improved by deepening the network and increasing the number of feature planes, making the parameters in the network increase greatly and the calculation of the network model more complicated. Therefore, the real-time detection efficiency of the network will be lowered.

At present, enterprises have realized product control under the two-dimensional development mode. However, how to realize the product control under the full three-dimensional mode is a key problem in industrial product control. DTs can provide a technical scheme for product control under the full three-dimensional mode. Therefore, the DT model is implemented in industrial product management and control, which confirms the importance of DTs. In addition, the efficiency of ultrasonic detection of internal defects in industrial production is improved, and an intelligent algorithm for automatic identification of internal defects is designed based on the relevant theory of lightweight deep learning. The algorithm has an excellent performance in ultrasonic defect detection of castings.

## 2. Materials and Methods

### 2.1. DTs Technology

DT is a simulation process that makes full use of the physical model, sensor update, operation history, and other data, integrates multidisciplinary, multiphysical quantity, multiscale, and multiprobability, and completes mapping in virtual space, to reflect the whole life cycle process of corresponding physical equipment. DTs can also be called digital images or digital mapping. DTs create a virtual model of the physical object in a digital way, to simulate the behavior of the physical object in the real environment [12–15]. One twin in the DTs is an entity that exists in the real world. This entity can refer to a part, such as a simple screw, or a factory, or even a complex human structure. The other twin in the DTs only exists in the virtual and digital world, which is the symmetrical mirror of the real world created by digital technology. It can map various attributes of physical equipment to the virtual space with the help of digital means such as design tools, simulation tools, the IoT, and virtual reality, to form a digital image [16, 17]. The DTs can be realized from different dimensions, as shown in Figure 1.

A typical DTs system usually includes physical objects, measurement perception, terminal controller, communication network, DTs operation platform, and user domain (Figure 2). These five parts are interrelated, which can achieve positive data acquisition and transmission analysis and realize reverse data feedback and decision control, forming a closed-loop interconnection of information transmission.

In general, DTs refers to a virtual model that is completely corresponding and consistent with the physical entities in the real world and can simulate its behavior and performance in the real environment in real time, also known as the DTs model [18, 19]. DTs are the key technology for manufacturing enterprises to move towards the strategic goal of Industry 4.0. It connects all stages (product creativity, design, manufacturing planning, production, and use) through the digital idea of mastering product information and its life cycle process and connects to production intelligent devices that can understand and respond to these pieces of information.  Figure 3 demonstrates the application of DTs technology in the equipment industry.

The corresponding functions of DTs technology in different stages are also different, as signified below.

#### 2.1.1. DTs in the Design Stage

In the product design stage, the accuracy of design can be greatly improved through DTs, and the performance of products in the real environment can be verified. The specific functions include digital model design, simulation, and imitation [20]. As for the product DTs, a model-based system-engineering-product development model will be developed driven by demand. It will realize the whole closed-loop management of “demand definition-system simulation-function design-logic design-physical design-design simulation-physical test.”

#### 2.1.2. DTs in the Manufacturing Stage

Building a virtual production line to meet manufacturing needs through digital methods requires a high degree of collaboration at this stage, and various factors such as products, equipment, production, and supervision need to be concentrated and coordinated.  Figure 4 demonstrates the implementation method, which mainly includes three functions. If some abnormal conditions that violate the strategy are found in the production process, these abnormal conditions need to be adjusted or handled in time to ensure the stability and optimization of the production process [21].

#### 2.1.3. DTs in the Service Stage

In recent years, the development of IoT technology has become gradually mature, accompanied by the corresponding reduction of the cost of sensors, not only large equipment but also some consumer products. These industrial products collect the working environment and state in the product operation stage through sensors and then analyze and optimize the collected information. This can both prevent faults in product production and help to improve the user experience of products [22].  Figure 5 illustrates the functions that DTs can achieve in the service phase.

The realization of remote monitoring and predictive maintenance function is to read the sensors of intelligent industrial products or various parameters of the control system. Then, remote monitoring is established, health evaluation indicators are built, and the prediction through AI is realized [23]. Next, the maintenance strategy is optimized according to the predicted results, to reduce the loss caused by unplanned downtime. The production index function of customers is optimized because many industrial customers realize production through industrial equipment. So, whether the setting of these industrial equipment parameters is reasonable and applicable to different production conditions is determined by the quality of customers' products and delivery cycle [24]. On the one hand, it can speed up the introduction cycle of new products, prevent some problems caused by the wrong use of products, and improve the accuracy of parameter configuration. On the other hand, obtaining the real needs of customers in this way can greatly reduce some mistakes in R&D decision-making [25].

### 2.2. Workench Simulation Platform

Workench is a collaborative simulation environment proposed by ANSYS company. Its user interface is more user-friendly than that of the classic ANSYS. Researchers can pay more attention to product R&D when using Workench. Furthermore, Workench can be well connected with SolidWorks software to import complex three-dimensional models into Workench simulation platform, which can solve the previous heterogeneous problem [26].

Under the environment of Workench and CAD collaborative simulation, all these steps can be completed on this platform, from product concept design to model simulation analysis and finally to the preliminary finalization of products, which greatly improves the work efficiency of designers. In the collaborative simulation environment, in addition to the sharing of Workench and various CAD software, hardware, and data resources, it can also allow different designers and analysts to carry out collaborative R&D, data integration, and data exchange, which will help to improve the efficiency of design R&D and shorten the design cycle [27].

### 2.3. Behavior Model Based on Finite State Machine

The behavior model of DTs refers to the geometric model driven by disturbance factors and driving factors, so that it has the behavior ability of response mechanism and physical entities and the ability of complex actions. That is, the response of geometric models is driven by multisource data of physical entities. Creating a physical production line behavior model is a complex process, so Moore finite state machine modeling method is used to create a production line system or device object behavior model. The finite state machine (FSM) is a mathematical model of the behavior of the system or object obtained abstractly. The mathematical model is a set of different states of the system or object. The multisource data set of the system equipment and the transition rules between states are used to describe the behavior process of the system or object. The FSM consists of three parts: all possible states of the system or object; the input set of the system or object, the input set received by the FSM in the process of motion; a set of rules for state transitions of a system or object. When a system or object receives different input information, the state of the machine changes from one state to another. Moore's classical finite state machine model is expressed as a six-tuple:

(1) $$\begin{array}{c} M=\left(Q,\sum ,\Delta ,\delta ,\lambda ,q_{0}\right). \end{array}$$

In equation (1), *Q*={*q*_0_, *q*_1_, *q*_2_,…, *q*_*n*_}, which indicates the set of finite states of the system or object can only be in a certain state during the movement;

∑={*δ*_0_, *δ*_1_, *δ*_2_,…, *δ*_*m*_} represents a finite input set of systems or objects;

Δ={*a*_0_, *a*_1_, *a*_2_,…, *a*_*r*_} denotes a finite input set of systems or objects;

*δ* : *Q* × ∑⟶*Q* refers to the state transition function;

*λ*⟶Δ represents the output function of the system or object, and the output function is only related to the current state of the system;

*q*_0_ ∈ *Q* stands for the initial state of the system or the object.

Equation (1) demonstrates that, in Moore FSM, the state of the next moment of state transition is determined by the current state and the current input state, and the output state is only determined by the current state, independent of the current input, and there is no state hesitating. Equation (1) is used to express defects existing in the production line behavior model. Improvements are made combined with the status of the intelligent processing production line as follows:

1. The output of Moore FSM only depends on the current state of the system or object, which is independent of the input at present, and there is *λ*⟶Δ. However, the real-time data of physical equipment throughout the production process is the engine for the system or object to make behavioral responses, so the output function of the production line should be determined by the current state of the system or object and the current real-time data; i.e., there is ∑×*λ*⟶Δ.
2. There is no “stop” state for the Moore FSM. However, in the actual production process, the production line has a state of shutdown and no movement, so the “stop” state *q*_*e*_ is added to the FSM.

Therefore, equation (2) illustrates the FSM model of the optimized intelligent processing production line.

(2) $$\begin{array}{c} \text{FSM}=\left(Q,\sum ,\Delta ,\delta ,\lambda ,q_{0},q_{e}\right). \end{array}$$

In equation (2), *Q*={*q*_0_, *q*_1_, *q*_2_,…, *q*_*n*_} indicates the set of finite states of the system or object, which can only be in a certain state during the movement;

∑={*δ*_0_, *δ*_1_, *δ*_2_,…, *δ*_*m*_} denotes the infinite input set of the system or the object;

Δ={*a*_0_, *a*_1_, *a*_2_,…, *a*_*r*_} represents the infinite output of the system or the object; *δ* : *Q* × ∑⟶*Q* stands for the state transition function;

∑×*λ*⟶Δ refers to the output function of a system or object, determined by the current state of the system or object and the current real-time data;

*q*_0_ ∈ *Q* bespeaks the initial state of the system or the object;

*q*_*e*_ ∈ *Q* accords with the final state of the system or the object.

Figure 6 indicates the working flow of the behavior model of the production line. Through the real-time data mapping module of the physical equipment of the production line, the real-time data of the production line system is mapped to the input set ∑={*δ*_0_, *δ*_1_, *δ*_2_,…, *δ*_*m*_} of the behavior model. The behavior model is calculated to output the behavior characteristics Δ={*a*_0_, *a*_1_, *a*_2_,…, *a*_*r*_} of the production line system. Then, the behavior characteristics and the internal logic of the equipment geometric model are combined to realize the behavior of the production line geometric model.

### 2.4. Establishment of Finite Element Model: Case Analysis

When the DTs of a product are established, the models of different working conditions and different scenes can be loaded on the DTs. One or more different DTs can be derived from each stage and each link, to carry out the simulation analysis, evaluation, and decision-making of various activities in the whole life cycle of the product, so that the physical products can obtain better manufacturability, assembly, detection, and security, as shown in Figure 7. The feasibility of the application of DTs in physics experiments is verified by case analysis.

#### 2.4.1. Element Selection and Mesh

Because the stress condition of each component of the aluminum alloy flange joint is complex, the geometric model of aluminum alloy flange is modeled by SolidWorks software and then imported into Workench simulation platform. High-order 3D 20 node solid structure element “Solid186” is adopted to ensure calculation accuracy. The high-order element is selected because it can simulate the boundary of the structural curve and surface, which is helpful to improve the calculation accuracy. However, when some structures with irregular shapes and uneven stress distribution are encountered, the high-order element can just avoid problems such as the shear locking.  Figure 8 manifests the flow of the finite element analysis.

Based on the high-order element “Solid186,” the mesh division at each irregular structure of the aluminum alloy flange node model is relatively fine. The purpose is to make the result of the stress concentration area more accurate. Simultaneously, the division scale of other parts of the flange node is relatively large, which is to reduce the computing resources of the node to a certain extent.  Figure 9 demonstrates the mesh of a specific element grid.

#### 2.4.2. Settings of the Contact Surface and Constitutive Model of Material

When the axial load acts on the flange joint, the nut ring, flange, screw, and cushion block will be in contact with each other. Except that the friction-free contact is set between the screw and the bolt hole, all other parts are set in friction contact, and the friction coefficient is 0.15. Sliding contact is automatically controlled. Fine sliding is adopted where rotation or sliding is relatively large, which can allow sliding or separation on the contact surface. Small sliding is used in other places, which can enhance the convergence and increase the calculation speed when the accuracy is guaranteed.  Table 1 lists the settings for the contact surface and the target surface, during the calculation of the contact pressure.

The components of aluminum alloy flange joints are assembled by extrusion and welding of aluminum alloy materials. Therefore, it is necessary to define the flange and the tube separately, and the Ramberg-Osgood model is used to define the constitutive model of the material, as shown in Figure 10. The nominal yield strengths *f*_0.2_ of aluminum alloy flange and aluminum alloy tube are 265.22 Mpa and 233.40 Mpa, respectively, and the ultimate tensile strengths are 292.71 Mpa and 252.82 Mpa, respectively. The fastener bolt is a 10.9-grade high-strength bolt, and its yield strength is 500 Mpa.

#### 2.4.3. Boundary Conditions and Assembly Settings

The setting of the boundary conditions of the finite element model remains the same as the actual test situation. One end of the specimen is fixed and constrained, and the other end is loaded with displacement control. The convergence is improved by turning on the weak springs switch in the workbench solution module. In the analysis, firstly, the bolt preload is applied, and then each contact pair is created. Secondly, the displacement load is applied after the bolt preload is locked until the joint is completely damaged.

### 2.5. Product Defect Identification and Detection

CNN is a change structure based on multilayer perceptron (MLP), proposed by Hubel and Wiesd in their early research on the primary visual cortex in the cat visual system. During the study, they found that the primary visual cortex of cats had two different cells, simple cells and complex cells. Through simple cells, special edge signals in the receptive field can be perceived, while the input of complex cells is the output of simple cells. In this way, the perception of edge stimulation signals can be realized in a larger receptive field [28]. CNN is actually a simulation of the biological visual cortex, which contains three unique structures: local receptive field, shared weight, and downsampling process, so that it can ensure the invariance of displacement, scaling, and distortion.

By using the local receptive field and weight sharing CNN, the feature image containing only some features can be extracted, which makes its translation invariant to the image, and CNN is not sensitive to locating the features [29]. At present, deep learning algorithms, especially CNN, are widely used in face recognition, natural language processing, general object recognition, robot, and automatic driving technology and have achieved very successful results [30]. The classical CNN structure generally includes an input layer, convolution layer, activation layer, pooling layer, fully connected layer, and output layer.  Figure 11 is a schematic diagram of the network structure.

The convolution layer is unique to CNN, and its activation function ReLU is expressed as follows:

(3) $$\begin{array}{c} \text{ReLU}\left(x\right)=\max\left(0,x\right). \end{array}$$

The characteristic calculation corresponding to the convolution layer is defined as follows:

(4) $$\begin{array}{c} y_{n}^{l}=f_{1}\left(\sum_{m\in V_{n}^{l}}y_{m}^{l-1}⊗\omega_{m,n}^{l}+b_{n}^{l}\right). \end{array}$$

In (4), *y*_*n*_^*l*^ is the nth characteristic graph in the *l*th layer, *b*_*n*_^*l*^ represents the offset value connected to the *l*th layer, *ω*_*m*,*n*_^*l*^ indicates the weight of the connection between the m-th characteristic graph in the upper layer of the *l*th layer and the nth neuron in the *l*th layer, and *V*_*n*_^*l*^ denotes the set of characteristic graphs connected to the *l*th layer.

Based on the basic theory of CNN, considering that the complexity of the picture itself is not particularly high and the amount of information is relatively small, it is designed to include a convolution layer, a pooling layer, and a fully connected layer. The output layer uses the Softmax function as the activation function and MATLAB software programming to realize the construction of the network. The Softmax function is a commonly used activation function in CNN, expressed as follows:

(5) $$\begin{array}{c} S_{j}=\frac{e_{j}^{x}}{\sum_{i=0}^{j}e_{i}^{x}}. \end{array}$$

However, the CNN model will become more and more complex with the network depth and the number of feature planes, the parameters in the network will increase greatly, and the amount of calculation of the network model will also increase. Hence, the real-time detection efficiency of the network will become low. Thus, based on deep separable convolution and channel shuffling, a lightweight CNN architecture is designed. Deep separable convolution factorizes the standard convolution method into deep convolution and point-by-point convolution. Deep convolution convolutes the input characteristic map channel by channel, and one convolution kernel is responsible for one channel. Each feature map obtained by deep convolution cannot contain all the information of the input feature map. Therefore, point-by-point convolution is used to carry out multichannel convolution again for the characteristic map output by deep convolution, so that the information can be retained as much as possible. Through deep separable convolution, the number of parameters of the model can be reduced while ensuring the smooth flow of information. The flow comparison of deep separable convolution and standard convolution is shown in Figure 12.

A new basic module of CNN is constructed by replacing 1 × 1 point-to-point convolution with group convolution and channel shuffling and then combined with the deep separable inversion residual convolution module, which is named Magnet. The overall structure of MagnetNets is a series of Magnet modules and some ordinary convolution layers. MagnetNets start with an input size of a standard volume layer, then stack with some Magnet modules, and then average pooling without any parameters. In the output of the last convolution layer, a fully connected layer is usually used as the input, but the number of parameters in the fully connected layer is very large, which may lead to overfitting and reduce the expression effect of the model. Therefore, the global average pooling is used to replace the fully connected layer, and a dropout layer is equipped to increase the network generalization ability to avoid overfitting. Finally, the output in the dropout layer is used as the input of the Softmax classifier to classify and detect the pictures.

ImageNet is a recognition project of the computer vision system, which is the largest database of image recognition in the world. The paper trains and tests the network models of MobileNets, ShuffleNet, Xception, MobileNetV2, and MagnetNets on the classified image data set of ImageNet. The TensorFlow framework is used to train the model, Xavier is used to initialize the parameters of the network model, and AdamOptimize is used as the optimization algorithm of the optimizer. Meantime, batch standardization is used after each layer. The batch size is 96 and the weight attenuation is 0.00004. The initial learning rate is set to 0.045, and the attenuation rate of the learning rate is 0.98 per generation. During the experiment, the data of internal defects of metal products are collected by manual detection, and a total of 110 defect-free images and 680 defect images are collected and processed by digital image technology. 90% of the data is used for training and 10% is used as test data to facilitate comparison and analysis. The data is input in random order, and the error in the training process is set to be less than 0.01.

## 3. Results and Discussion

### 3.1. Comparative Analysis of Finite Element Analysis Results and Test Results

#### 3.1.1. Deformation Mechanism and Failure Mode

Figure 13 displays the stress nephogram of failure mode obtained by simulation of the specimen.

Figure 13(a) reveals that the deformation mechanism and failure of the finite element simulation of the FL164 specimen are basically the same as those of the test, and the radial shrinkage failure occurs at the connection between the stiffener and the circular tube.  Figure 13(b) indicates that, in the tensile process, besides the large deformation of aluminum alloy circular pipe, when the node is in failure, the stiffener has a relative buckling, which is consistent with the test results.  Figure 13(c) demonstrates that when the flange is disassembled for axial tension, there is no obvious deformation or warpage of the flange plate, and the dent of the cushion block is obvious.  Figure 13(d) signifies that the top of the high-strength bolt also has a diameter shrinkage phenomenon. The inner side of the bolt is under tension and the outer side is under pressure, which is the same as the test phenomenon.

#### 3.1.2. Development Trend of Finite Element Stress Simulation

When the test piece FL164 is subjected to the ultimate load, firstly, the aluminum alloy round pipe shrinks, secondly, the bolt slides, and thirdly, the heat-affected zone of the weld breaks.  Figure 14 presents the failure characteristics of the test piece at this time.

Figure 14 demonstrates that the stress on the aluminum alloy round pipe is relatively large, so the diameter shrinkage occurs. The corresponding diameter shrinkage phenomenon also appeared at the uppermost part of the screw, while the thread sliding phenomenon appears in the thread area at the lower end of the bolt. The dent at the orifice on the cushion block is obvious, and the phenomenon of stress concentration appears. During the tensile process of the specimen, the weld joint appears to tumble to a certain extent, and the fracture occurs at the position of the welded heat-affected zone.

The specific stress analysis of the FL164 flange joint is carried out, and Figures 15–17 demonstrate the stress development process of the specimen. That is, firstly, the aluminum alloy round pipe shrinks; secondly, the bolt slides; thirdly, the heat-affected zone of the weld breaks. The trend of stress development is basically consistent with the test.

Figure 15 indicates that when the load is close to the yield load, the place where the aluminum alloy round pipe is connected with the end of the stiffener begins to yield, the middle and top parts of the aluminum alloy round pipe are still in the elastic state, and the stress state of the screw changes from the tensile force to the tensile bending state due to the large internal stress.

Figure 16 indicates that when the aluminum alloy circular pipe enters the full section yield, the welding part of the stiffener begins to yield, so it is subjected to a relatively large stress, while the flange is still in an elastic state, and its safety margin is relatively large.

Figure 17 implies that when the position of each node of the flange fails, the overall yield of the aluminum alloy circular pipe will be caused, and the welding part of the stiffener will be subjected to great stress, but the flange is still in an elastic state.

From the above analysis, the conclusion is that the nonlinear finite element analysis can well analyze the stress change process and failure state of the joint, which is highly consistent with the tensile process of the test axis. Therefore, it can be proved that the finite element analysis method is relatively reliable.

### 3.2. Load-Displacement Curve

Figure 18 demonstrates the test load-displacement curves of two groups of specimens.

Figure 18 bespeaks that the test load-displacement curve of the FL164 specimen is well consistent with the finite element results. The finite element analysis method can simulate the ultimate load and yield load of the joint. However, in the beginning, the stiffness of the finite element analysis result is larger than that of the test result. This is mainly because the finite element models are carried out under ideal conditions.

### 3.3. Comparison Results of Network Models

The experimental results and the data compared with other network models are shown in Figure 19.

Figure 19 shows that the accuracy of the designed lightweight CNN is 94.1% and the size of the model is 2.9 MB. The accuracy of MagnetNets is as high as that of MobileNetV2 and other network models. And MagnetNets' weight is lighter than others.

### 3.4. Defect Identification Test Results of CNN

Import the prepared test data into the MagnetNets network model to verify the training effect. The test results are shown in Figure 20.

As Figure 20 reflects, the detection accuracy of the MagnetNets network model is very high. MagnetNets network model has great advantages in ultrasonic defect recognition. The six experiments reveal that the MagnetNets network model shows stable performance. MagnetNets network model has a very good effect on image feature extraction and learning. With sufficient training, it can achieve 100% recognition accuracy. The above experiments conclude that the MagnetNets network model has an excellent performance in ultrasonic defect detection of castings.

## 4. Discussion

Under the traditional research and design mode, paper and 3D CAD are the main product design tools. The virtual model established by them is static, and the change of physical objects cannot be reflected in the model in real time, nor can it be communicated with the product life cycle data such as raw materials, sales, market, and supply chain. In the technical verification of new products, it is necessary to produce the products and conduct repeated physical experiments to obtain limited data. The traditional R&D design has the characteristics of a long cycle and high cost.

DT breaks through the limitations of physical conditions, helps users understand the actual performance of products, and iterates products and technologies with less cost and faster speed. DTs technology supports three-dimensional modeling, realizes paperless parts design and assembly design, and replaces the traditional way of obtaining experimental data through physical experiments. Virtual experiments are carried out by means of calculation, simulation, analysis, and so on, to guide, simplify, reduce, or even cancel physical experiments.

Users use structural, thermal, electromagnetic, fluid, and control simulation software to simulate the operation of the product and test, verify, and optimize the product. With the upgrading of industrial products from mechanization to multidisciplinary integration, informatization, and networking, the timeliness, systematicness, and comprehensiveness of experimental verification are facing great challenges. The verification based on physical tests is limited by the development cycle, cost, and environmental conditions. The sample is limited and it is difficult to completely cover the limit deviation combination state. As a new technical approach, the virtual test has the advantages of the short cycle and low cost, which can easily carry out the test types that are difficult to be carried out by physical objects such as limit condition test and fault test. In engineering practice, according to the accuracy of the virtual test and the perfection of system, give full play to the advantages of physical test and virtual test, virtual and real integration, and complimentary promotion and improve the comprehensive testability of products.

## 5. Conclusion

So far, DTs have been successfully applied to different industries, including product design, production, prediction, health management, and other fields. Based on the application of DTs technology in industrial product management and control, and taking the DTs in the design stage of industrial product management and control as the research object, this paper connects Workench simulation platform and SolidWorks software and applies it to the design of aluminum alloy flange. Through the comparison of the results of the test and simulation, the present work confirms the role of DTs in industrial product management and control. The results show that the nonlinear finite element analysis results are well consistent with the experimental results and contribute to the improvement of design R&D efficiency and the shortening of the design cycle. MagnetNets network model has an excellent performance in ultrasonic defect detection of castings. DTs break through the limitation of physical conditions, help users understand the actual performance of products, and iterate products and technologies with less cost and faster speed. The deficiency is that, due to the limited time, the study is only conducted for the DTs in the design stage of industrial product management and control, but without the application of DTs in the whole process of industrial product management and control. Therefore, more research will be carried out in this aspect in the future. In addition, the defect is recognized by learning ultrasonic image data, but more specific defects can be detected through CNN, and the size of defects can be identified by learning.

## Figures and Tables

**Figure 1:** Implementation form of different dimensions of DTs.

**Figure 2:** Architecture of DTs system.

**Figure 3:** Application of DTs technology in the equipment industry.

**Figure 4:** Functions realized by DTs in the manufacturing stage.

**Figure 5:** Functions of DTs implementation in service stage.

**Figure 6:** Behavior model.

**Figure 7:** Application scene of the DTs in the product reliability.

**Figure 8:** The flow of the finite element analysis.

**Figure 9:** The meshing of the joint.

**Figure 10:** Material constitutive model.

**Figure 11:** CNN structure diagram.

**Figure 12:** A process comparison between DSC and standard convolution.

**Figure 13:** Stress nephogram of failure mode. (a) FL164 overall stress nephogram, (b) weld rolling, (c) cushion block dent, and (d) bolt tension bending.

**Figure 14:** Failure characteristics of the test piece. (a) Circular shrinkage fracture. (b) Bolt diameter reduction sliding wire. (c) Cushion block hole dent. (d) Heat-affected zone fracture.

**Figure 15:** Stress nephogram of initial yield. (a) Aluminum alloy round pipe. (b) Stiffener welds. (c) Bolt.

**Figure 16:** Stress nephogram at partial “full section yield.” (a) Aluminum alloy round pipe. (b) Stiffener welds. (c) Bolt.

**Figure 17:** Stress nephogram of specimen failure. (a) Aluminum alloy round pipe. (b) Stiffener welds. (c) Bolt.

**Figure 18:** Load-displacement verification diagram.

**Figure 19:** Comparison results of various network models.

**Figure 20:** CNN test results.

**Table 1:** Contact settings of flange nodes.

Number	Contact type	Target surface	Interface

1	Face-to-face contact	Stainless steel flange	Nut torus
2	Face-to-face contact	Stainless steel flange	Aluminum alloy flange
3	Face-to-face contact	Q235 cushion block	Aluminum alloy flange
4	Face-to-face contact	Q235 cushion block	Nut torus
5	Face-to-face contact	Q235 cushion block hole	Screw
6	Face-to-face contact	Flange hole	Screw

## Data Availability

The data used to support the findings of this study are included within the article.
